The article "The Four Pillars for Successful Regenerative Therapy in Endodontics: Stem Cells, Biomaterials, Growth Factors, and Their Synergistic Interactions" was published in 2022. Journal: Stem Cells Int.

# The Four Pillars for Successful Regenerative Therapy in Endodontics: Stem Cells, Biomaterials, Growth Factors, and Their Synergistic Interactions

**DOI:** 10.1155/2022/1580842

**Published:** 2022-09-19

**Authors:** C. Brizuela, George T.-J. Huang, A. Diogenes, T. Botero, M. Khoury

**Affiliations:** ^1^Facultad de Odontología, Universidad de Los Andes, Santiago, Chile; ^2^School of Dentistry, The University of Tennessee Health Science Center, Memphis, USA; ^3^School of Dentistry UT Health San Antonio, San Antonio, USA; ^4^School of Dentistry University of Michigan, Ann Arbor, USA; ^5^Laboratory of Nano-regenerative Medicine, Faculty of Medicine, Universidad de los Andes, Santiago, Chile; ^6^Cells for Cells, Regenero, Santiago, Chile; ^7^IMPACT, Center of Interventional Medicine for Precision and Advanced Cellular Therapy, Santiago, Chile

## Abstract

Endodontics has made significant progress in regenerative approaches in recent years, thanks to advances in biologically based procedures or regenerative endodontic therapy (RET). In recent years, our profession has witnessed a clear conceptual shift in this therapy. RET was initially based on a blood clot induced by apical bleeding without harvesting the patient's cells or cell-free RET. Later, the RET encompassed the three principles of tissue engineering, stromal/stem cells, scaffolds, and growth factors, aiming for the regeneration of a functional dentin pulp complex. The regenerated dental pulp will recover the protective mechanisms including innate immunity, tertiary dentin formation, and pain sensitivity. This comprehensive review covers the basic knowledge and practical information for translational applications of stem cell-based RET and tissue engineering procedures for the regeneration of dental pulp. It will also provide overall information on the emerging technologies in biological and synthetic matrices, biomaterials, and signaling molecules, recent advances in stem cell therapy, and updated experimental results. This review brings useful and timely clinical evidence for practitioners to understand the challenges faced for a successful cell-based RET and the importance of preserving or reestablishing tooth vitality. The clinical translation of these current bioengineering approaches will undoubtedly be beneficial to the future practice of endodontics.

## 1. Introduction

Regenerative endodontic concept was brought to attention in the 2000s when several case reports were published showing without apexification procedures, immature tooth apex appeared to mature while the lesion healed. They used sodium hypochlorite (NaOCl) irrigation and triple-antibiotic paste within the root canal, followed by induction of bleeding through apical tissue laceration and blood clot formation inside the root canal [1].

The article "The Four Pillars for Successful Regenerative Therapy in Endodontics: Stem Cells, Biomaterials, Growth Factors, and Their Synergistic Interactions" was published in 2022. Journal: Stem Cells Int.

It was thought that the blood clot may work as a matrix for mesenchymal stem/stromal cell (MSC) migration from periapical tissue into the root canal. Murray et al. called for the significance of regenerative approach for endodontic treatments, and the term “regenerative endodontics” was advocated [2].

As well as blood clots, autologous platelet-rich plasma (PRP) and platelet-rich fibrin (PRF) have also been introduced into the root canal as alternative scaffolds because platelet-derived products contain molecules that can induce pulp-dentin regeneration [3–5].

Subsequently, more cases have used the bleeding technique but with different irrigation or medication with successful resolution of apical periodontitis, promoting continuous root development and revitalization of pulpless teeth ([6], de Jesus Soares et al. [7], Gelman et al. [8], Mccabe et al. [9, 10]).

Regenerative endodontic therapy (RET) aims to regenerate the pulp-dentin complex damaged by infection, trauma, or developmental anomaly of immature permanent teeth with necrotic pulp [11].

Recent evidence points at the possibility of bringing vital tissues into the damaged pulp through the application of three main components: stem cells, signaling molecules, and a physical scaffold that can support cell growth and differentiation [12]. The synergistic effect of these elements promotes the reparative potential of resident cells within the pulp and concurrently and enhances the migration capacity of the recipient's stem cells toward the injury site [13].

To enhance the possibility of pulp-dentin regeneration, different interventional advanced approaches are required. There are two different approaches to perform RETs [14]. That is either cell-free (CF)-RETs that attempt to induce host endogenous cells or stem cells migrate into the root canal for regeneration or cell-based (CB)-RETs which introduce exogenously prepared cells or stem cells into the canal for regeneration. CB-RET incorporates undifferentiated MSCs or pulp MSCs into the root canal, which can be differentiated into an odontoblast phenotype and synthesize pulp-dentin matrix. CB-RET offers many advantages compared with cell-free RETs because it has control over the factors that could initiate true pulp-dentin regeneration (Table 1) in contrast to cell-free RET (CF-RET). For example, CB-RET potentially manage the amount, nature, and age of the cells participating in the process, and it can use allogenic MSCs in elderly patients. There is substantial interest in applying allogenic MSCs, because autologous MSCs have limited sources and there is a need for off-the-shelf immediate availability for cell therapy [15, 16]. CB-RET allows clinicians to select the most suitable scaffold (biological or synthetic) for successful results and uses additional growth factors to modulate transplanted MSCs or autologous MSCs in pulp-dentin regeneration.

The article "The Four Pillars for Successful Regenerative Therapy in Endodontics: Stem Cells, Biomaterials, Growth Factors, and Their Synergistic Interactions" was published in 2022. Journal: Stem Cells Int.

In this review, we bring together the multidisciplinary facets required for the application of scientifically proven RET. The discussion of future perspectives and challenges would orient clinicians to form a critical, consensual, and objective opinion leading to a better understanding of this emerging field.

## 2. Review

### 2.1. First Pillar: Stem Cells and Pulp Regeneration

#### 2.1.1. The Goal of Pulp Regeneration

The goal of tissue regeneration is to regenerate the lost or damaged tissue or organ to its original state [17]. The regenerated tissue should be functional and seamlessly integrated into the adjacent tissues. The same principle is applied to the field of regenerative endodontics [18]. Previously, Huang and colleagues have discussed pulp regeneration by recognizing a critical concept in tissue engineering. That is, using stem cell-based (CB-RET) or cell-free approach (CF-RET) to categorize pulp-dentin regeneration [19, 20]. CB-RET is defined as delivering exogenously prepared cells, often cultured in vitro, into the host for tissue regeneration, whereas CF-RET does not deliver any exogenous cells into the host but relies on endogenous cells for the regeneration [14] (Figure 1).

Comparison between CF-RET and CB-RET are in Table 1. CF-RET has not generally shown to regenerate pulp or dentin, but periapical tissues including cementum, bone, and periodontal ligament grow into the canal space [21].

#### 2.1.2. Dental Stem Cells for Pulp Regeneration

The stem cells used for pulp regeneration for animal models or human trials have been from pulp or apical papilla, including dental pulp stem cells (DPSCs) from permanent teeth or stem cells of the exfoliated deciduous teeth (SHED) and stem cells from the apical papilla (SCAP) [22]. Most pulp regeneration studies used a heterogeneous population of DPSCs. In a dog model, subpopulations (SP) of DPSCs that are CD31- and CD105+ cells, showing angiogenic/vasculogenic and neurogenic potential suited for pulp regeneration [23]. The use of granulocyte colony stimulating factor (G-CSF) was shown to mobilized dog a DPSC subpopulation (MDPSCs) that contains high levels of CD105. These cells have also been shown to be a promising cell source for pulp regeneration, including for mature teeth with small apical foramen size of ~0.5 mm [24].

#### 2.1.3. Nondental Stem Cells for Pulp Regeneration

Although DPSCs or SCAP have been shown to be promising cells for pulp regeneration, the availability of autologous sources for these cells is limited, particularly in fully formed mature teeth. The more widely available nondental stem cells have been tested for their potential for dentin/pulp regeneration, bone marrow mesenchymal/stromal stem cells (BMSCs), or adipose tissue-derived stem cells (ADSCs) the primary nondental stem cells for these applications. In a dog orthotopic pulp regeneration model, G-CSF induced mobilization of canine DPSCs, BMSCs, and ADSCs, and these cells were able to form pulp-like tissue in the dog [25]. However, there was no convincing demonstration of dentin-like formation that was presented using these nondental stem cells. Notably, recently a human clinical trial using umbilical cord MSCs (UC-MSCs) has been reported with acceptable clinical outcomes such as the resolution of the infection, healing of the disease, continued radiographic root development, and reestablishment of vascularity and responses to the sensitivity testing [26]. Despite these promising clinical outcomes, the tissue formed by these procedures has not yet been characterized as full reestablishment of the pulp-dentin complex in its native form.

The article "The Four Pillars for Successful Regenerative Therapy in Endodontics: Stem Cells, Biomaterials, Growth Factors, and Their Synergistic Interactions" was published in 2022. Journal: Stem Cells Int.

### 2.2. Second Pillar: Biomaterials as Support for Cell Transplantation

In the search for proper pulp-dentin regeneration, several *in vitro* and *in vivo* models (Table 2) have been developed using different autologous or allogenic MSCs, natural or synthetic scaffolds, and different growth factors. Another hurdle is to secure an adequate blood supply for the survival of transplanted cells to ensure their regenerative potential [27]. Enhanced neovascularization is needed for more successful complete pulp regeneration especially if dealing with small canals. Tooth with large apical opening as shown in the tooth fragment mouse models, neovascularization is not an issue [28]. When the apex is smaller, and canal is longer and narrower, complete pulp regeneration is close to impossible without enhanced neovascularization as well discussed by Huang et al. and Nakashima et al. [22, 29]. The goal is to provide a suitable environment for cellular infiltration, proliferation, and differentiation [30]. To find new strategies for CB-RET, different scaffolding systems have been evaluated: (a) Restylane, a commercially available hyaluronic acid hydrogel [31], (b) microspheres with growth factors [32], (c) drug-loaded fiber with a vascular endothelial growth factor that stimulates angiogenesis and vasculogenesis [33], (d) nanofibrous poly(l-lactic acid) scaffolds and addition of simvastatin to evaluate anti-inflammatory, odontogenic, and proangiogenic effects on dental pulp cells (DPCs), which could be promising for dentin regeneration with inflamed dental pulp tissue, increasing the regenerative potential of resident stem cells [34], or (e) potential applications of polycaprolactone/submicron bioactive glass hybrid composites for pulp and dentin tissue regeneration, where DPCs have significantly higher proliferation and generate more mineralized nodules [35]. A class of smart material, such as phosphorene, has been introduced into medicine for various applications [36]. 2D sheets of black phosphorus called black phosphorene have been shown to serve as a scaffold to enhance bone regeneration [29]. Such materials may be worthy of investigation for their potential in pulp-dentin [36]. ECM-based scaffolds have shown promising results in terms of progenitor cell recruitment, promotion of constructive remodeling, and modulation of host responses; this makes them ideal candidates for pulp regenerative therapy and to support cellular infiltration [30].

The article "The Four Pillars for Successful Regenerative Therapy in Endodontics: Stem Cells, Biomaterials, Growth Factors, and Their Synergistic Interactions" was published in 2022. Journal: Stem Cells Int.

The use of scaffolds increases the risk of inflammation and infection [37]. Therefore, Dissanayaka et al. analyzed scaffold-free prevascularized microtissue spheroids containing DPCs and endothelial cells and then used scaffold-free microtissue spheroids of DPSCs prevascularized by human umbilical vein endothelial cells. These were inserted into the canal space of tooth root slices and implanted subcutaneously into immunodeficient mice, which resulted in well vascularized and cellular pulp-like tissues of human origin [27]. Interactions between endothelial and progenitor/stem cells are important for vascularization of regenerating tissue; thus, different scaffold, cells, and growth factors have been investigated for triggering angiogenesis and regenerating vascularized pulp, such as the peptide hydrogel PuraMatrix™ without growth factors [38] Figure 1.

### 2.3. Third Pillar: Effect of Cell-Derived Soluble Factors on Cell Homing and Resident Cells

Stem cells and their derived soluble bioactive factors are an important part of the triad of tissue engineering [39]. The fate of endogenous undifferentiated cells homed into empty root canal spaces from the apical tissues in CF-RET or by transplanting exogenously expanded cells in CB-RET is intimately associated with the molecular cues present in the microenvironment. These cues can be originating from a blood clot [40] or in blood-derived by-products such as platelet-rich plasma (PRP) or platelet-rich fibrin (PRF) that can be used as scaffolds and contain high concentrations of multiple growth factors. Notably, MSCs have been shown to exert potent paracrine effects by the release of growth factors that act on nearby cells, orchestrating their significant cellular response in the promotion of the regenerative process [41]. The release of these factors is modulated and increased particularly when placed in hostile environment such as a previously infected root canal where there is inflammation, residual microbial antigens, and hypoxia due to the lack of collateral circulation [42]. Collectively, many molecules have been identified and studied for their ability to promote cell homing, survival, proliferation, migration, and differentiation of MSCs. The process of cell homing is a specific physiologic event closely related to routine wound healing following injury [43] when cells are attracted to a region of injury requiring repair or regeneration. Numerous chemotactic factors have been identified in mammals. For example, the safety and feasibility of using granulocyte colony stimulating factor (G-CSF) in endodontic regeneration tested in preclinical studies formed the foundational knowledge for its application in a cell-based clinical trial in Japan [44] Similarly, fibroblast growth factor-2 (FGF-2) and stromal derived factor-1 (SDF-1) have been shown to be potent chemotactic factors and promote cell homing in vitro and in vivo studies [45, 46].

The article "The Four Pillars for Successful Regenerative Therapy in Endodontics: Stem Cells, Biomaterials, Growth Factors, and Their Synergistic Interactions" was published in 2022. Journal: Stem Cells Int.

### 2.4. Fourth Pillar: De Novo Interaction between Stem Cells, Biomaterials, and the Regenerative Milieu

The stem cell niche typically has a spatial organization that provides anatomical and functional interactions contributing to cell fate specification as well as the maintenance of their stemness potential (Sari [47]). These interactions are mutual and dynamic, including both cellular and acellular components. The critical constituent of the physiological milieu includes the following: (a) cellular counterparts (immune/inflammatory cells, perivascular and endothelial cells, and mesenchymal and stromal support cells, among others), (b) extracellular matrices including adhesion and signaling receptors, and (c) soluble factors (chemokines, hormones, and growth factors). Endogenous niche-directed interventions might be employed to boost support for stem cells in the case where they are transplanted without a scaffold or supportive factors. In a contrasting approach, the transplantation of cells, scaffold, and factors, part of the three pillars of regeneration mentioned above, constitute a controllable strategy to recapitulate the physiological stem cell niche. The understanding of the cellular players and molecular signals that constitute stem cell niches under different physiological but also pathological conditions are important cues to consider when developing ex vivo transplants that mimic with high fidelity their native environment. The adequate interaction between the expanded cells and their ex vivo engineered niche can predict their activities to promote tissue regeneration in vivo. Moreover, the synergy between all the constituent of the transplanted tissue on one hand and the interaction with the host environment will dictate the success or failure of the clinical intervention.

The article "The Four Pillars for Successful Regenerative Therapy in Endodontics: Stem Cells, Biomaterials, Growth Factors, and Their Synergistic Interactions" was published in 2022. Journal: Stem Cells Int.

#### 2.4.1. Strategy on Neovascularization during Pulp Regeneration

Currently, most pulp regeneration studies focus on large diameter canal spaces with short roots.

However, the challenge of developing an adequate vasculature is substantially more significant when considering smaller diameter canals with long roots since the coronal end of the canal space will be further away from the existing apical vasculature [48]. Thus, the engineered vasculature incorporated into pulp regeneration becomes critically important if to achieve a high level of success [29]. Rapid establishment of blood supply for the transplanted stem cells may be achieved by integrating engineered vasculature, often combined with a scaffold, which is critically important for those cells' survival [49].

Most currently employed RET protocols include creating intracanal bleeding to transfer undifferentiated progenitor cells from the apical region into the canal space and establish a scaffold harboring growth factor [50]. Indeed, this step has been shown to deliver substantial numbers of MSCs that far exceeds that of circulating systemic blood in both immature teeth in young individuals [51] and mature teeth in adults [52].

It is well-established that proper root development requires an intimate relationship between Hertwig's epithelial root sheath (HERS) and the undifferentiated cells of the apical papilla in immature teeth. The integrity of this critical interaction dictates root development and shape as damage of the HERS can result in the formation of roots with odd shapes and blunted apices, absence of root development [53], or formation of an apical root development that is not continuous with the main roots structure [54].

Considering the HERS' importance for continued root development, clinicians must be thoughtful when evoking the bleeding from the surrounding apical tissues while minimizing HERS damage. Alternatively, autologous blood by-products such as PRP and PRF have been used in multiple published cases to minimize the need for vigorous mechanical disruption of apical tissues. Nonetheless, minimal bleeding has been still evoked in most cases that use PRP or PRF, and even in 2 of the cell-based regenerative endodontic clinical trials that included transplantation of stem cells [26, 55].

The article "The Four Pillars for Successful Regenerative Therapy in Endodontics: Stem Cells, Biomaterials, Growth Factors, and Their Synergistic Interactions" was published in 2022. Journal: Stem Cells Int.

In addition to the clinical challenging of evoking sufficient blood to fill the root canal while not damaging the very structures responsible for root development, the delivery of cells to a pulpless root canal space poses many challenges. The primary challenge is delivering many heterogeneous cells to the canal space that is devoid of vascularity. Ideally, cells would progressively ingress into the root canal space using a suitable scaffold concomitant to develop supportive vascularity from the apical region to the coronal-most region of the root canal system. Instead, cells become trapped in the blood clot scaffold in a largely hypoxic environment. This hypoxic gradient has been shown to induce the expression and release of several proangiogenic factors from this cell [38]. This is likely an important factor that allows the newly formed tissues in RETs to become vascularized. Relatively fast angiogenesis has been demonstrated in the histological analysis of clinical cases of following RETs with vascularity seen as little as 3.5 weeks following treatment [56].

The transplantation of well-defined populations of stem cells expanded in culture has several advantages, including the introduction of homogenous high concentration of cells encapsulated in design scaffolds. This approach has been employed in clinical trials using a cell-based approach with transplantation of either DPSCs [44], autologous cells of deciduous teeth [55], or allogenic umbilical stem cells [26] in which cells were transplanted to the canals for pulp regeneration.

Despite the many advantages of the cell-based approach in regenerative endodontics, many barriers still need to be addressed before its widespread acceptance and use. An important issue is the effectiveness versus efficacy [57] compared to currently employed CF-RETs. Unfortunately, no comparative studies are evaluating successful clinical outcomes between CB-RET and CF-RET approaches in endodontics. Given that currently, cell-free approaches have been shown to result in high clinical successful outcomes, the rationale for a much more sophisticated cell-based approach must hinge on hypothesized improved predictability of results and the formation of a better organized pulp-dentin complex. However, there is minimal evidence that this approach does indeed result in full regeneration of the pulp-dentin complex, with only one case demonstrating the presence of a well-organized tissue with odontoblastic-like cells lining the canal walls [55].

### 2.5. Published Randomized Clinical Trials

Several studies in regenerative endodontics have been published, but still, there is a limited number of randomized clinical trials (Table 3). The evidence is relatively weak, and the probability of success depends on multiple conditions found in individual cases. This knowledge gap is influenced by the enormous diversity of protocols [58], making the predictability of these therapies uncertain [23]. The most recent and comprehensive randomized clinical trial in regenerative endodontics was published by a group of investigators from China, Lin et al. in 2017 [59]. The authors concluded and confirmed results from previous retrospective and prospective case series studies; they found how the etiology has impacted the outcome. CF-RET and apexification can achieve the primary goal, elimination of symptoms, and evidence of bone healing, but the secondary outcome of continuation of root development and tertiary outcome of evidence of pulp vitality were only found with the cases treated with CF-RETs [59].

The article "The Four Pillars for Successful Regenerative Therapy in Endodontics: Stem Cells, Biomaterials, Growth Factors, and Their Synergistic Interactions" was published in 2022. Journal: Stem Cells Int.

The control of the infection established in the root canal and periapical tissues is critical [60]. However, it is also essential to preserve the stem cells' vitality present on the apical papilla. Nevertheless, the control of microorganism reinfection is crucial to regenerate the dentin-pulp complex [60]. Even with the infection under control, there are still challenges, such as creating a blood clot as a scaffold and preserving the apical tissue's regenerative potential. Innovative research and its clinical application have been done to overcome these challenges by introducing platelet-rich plasma and platelet-rich fibrin scaffolds (PRP and PRF) [61–63] to induce in situ stem cell proliferation or cell homing protocols. However, still, not much difference in outcomes has been found [3, 64, 65].

Histologically, most in vivo studies and isolated case reports have demonstrated periodontal tissue in growth in the canal space, including bone, cementum, and a fibrous connective tissue, instead of a pulp-dentin complex. This reparative process has been termed guided endodontic repair [66], whether the stem cells might be predominantly from the bone marrow or the periodontal ligament, still to be demonstrated. Researchers have focused efforts on implanting stem cells in the root canal to ensure more predictable healing. Although most studies have been conducted in vitro and in vivo animal models [44], a recent demonstration of this approach's feasibility in patients has been published by Dr. Nakashima and colleagues in Japan [67]. This pioneer pilot study of autologous stem cell transplantation into mature human teeth demonstrated the feasibility of stem cell therapy in endodontics. A more extensive clinical trial of autologous stem cell transplantation into immature human teeth reported by Drs. Shi and Jin and colleagues further validated a promising future for stem cell-mediated therapy in endodontics [55]. Research on the pulp-dentin complex's regeneration requires applying tissue engineering concepts with controlled delivery of the appropriate cells, growth factors/morphogens, and scaffolds, unlike a revascularization (CF-RET) protocol, where evoked bleeding is thought to be sufficient for reestablishment of function and acceptable clinical outcomes.

The article "The Four Pillars for Successful Regenerative Therapy in Endodontics: Stem Cells, Biomaterials, Growth Factors, and Their Synergistic Interactions" was published in 2022. Journal: Stem Cells Int.

More evidence is needed from comparative well-controlled studies evaluating efficacy and from additional studies performed in clinical practices to investigate the “real-world” application of this approach and evaluate its effectiveness in the hands of practicing clinicians. In summary, further studies warrant improving cell-free therapies that already presently benefit patients and allow the transition of cell-based approached from very few well-controlled university-based studies [26, 44, 55] to clinical practices.

### 2.6. Challenges and Future Perspectives

Considerable effort has been made for the regeneration of the dental pulp; however, the newly formed tissue has not been yet characterized as full reestablishment of the pulp-dentin complex in its native form. This attribute is very important for determining whether the outcome can be defined as the repair of the tissue architecture and function or the regeneration referring as the completely restoration of damaged tissue to their normal state.

While these adult stem cells including MSCs have varying differentiation and transdifferentiation ability, pluripotent stem cells, such as embryonic stem cells (ESCs) and induced pluripotent stem cells (iPSCs), have unambiguous potential for differentiation into multiple lineages [68]. Most important, these pluripotent stem cells can self-renew indefinitely as an unlimited cell source for tissue regeneration. As a result, their differentiation to the various cell types of cells including MSCs [69] could be considered to be one of the most promising cell sources for dental pulp regeneration.

The histological characterization has not fully differentiated all standard features of odontoblasts, and there was no evidence of tubular dentin formation in the reported case that represented only one sample of the cases included in this clinical trial [70]. Perhaps some of the confusion of what constitutes an acceptable presentation of proper pulp regeneration lies in the insufficient consensus of the evaluated criteria. Also, the evidence of desirable histological outcomes shown in animal models of pulp regeneration is based on sterile models in the absence of inflammation [71].

The article "The Four Pillars for Successful Regenerative Therapy in Endodontics: Stem Cells, Biomaterials, Growth Factors, and Their Synergistic Interactions" was published in 2022. Journal: Stem Cells Int.

Another important challenge is to achieve a correct disinfection of the root canal system; the literature has shown that this aspect is very necessary to achieve the success of regenerative therapies. Infection models have been tested in large animal systems in CF-RET and CB-RET studies and demonstrate that residual bacteria have a critical negative effect on the outcome of regenerative endodontic procedures. Some study demonstrates in a CF-RET model that there were no differences among the medicaments investigated in radiologic treatment outcomes, but disinfectants in REPs showed altered microbiota from normal and diseased immature teeth with different histologic patterns of regeneration [72]. Also, Verma et al. showed CB-RET model that the presence of residual bacteria is a major risk to the success of regenerative procedures [60].

For promoting expectable pulp-dentin regeneration, optimum antimicrobial approaches need to be developed for appropriate disinfection of infected roots while guaranteeing survival, recruitment, proliferation, and differentiation for CF-RET and CB-RET. The latest improvements in scaffold-free therapy include the use of extracellular vesicles (EVs) released from stem cells. MSC-derived EVs show potent proangiogenic and immunomodulatory effects that have been investigated in various inflammatory diseases [73].

Recently, EVs isolated from DPSCs were shown to promote angiogenesis in an injectable hydrogel in vitro, offering a novel and minimally invasive strategy for regenerative endodontic therapy [74]. The cargo carried by DPSC-derived exosomes, which may have various effects on bone tissue formation, is thought to vary depending on the culture conditions and donors which can lead to different clinical outcome. Further studies on the DPSC cargo and the effects of high doses and concentrations of exosomes are needed before using EVs in endodontic procedures [74].

Beside EVs, the effects of mitochondrial transfer have surfaced as a new cell-free approach for the treatment of inflammatory diseases [75]. In addition, mitochondrial exchange is currently being considered as one emerging mechanism of action through which MSCs can be beneficial for multiple cellular processes [76], such as graft versus host disease [77] and sepsis to regenerate and repair damaged cells or tissues [78]. It has been evident that this transfer is a major key in immune regulation, healing several diseases related to brain injury, cardiac myopathies, muscle sepsis, lung disorders, and acute respiratory disorders that can be also applied to dental condition where inflammation plays an important trigger role [79]. Both EVs and mitochondria transfer technologies represent good examples of future applications to be delivered alone or in combination of the different approaches mentioned above such as stem cell-derived factors and biomaterials.

The article "The Four Pillars for Successful Regenerative Therapy in Endodontics: Stem Cells, Biomaterials, Growth Factors, and Their Synergistic Interactions" was published in 2022. Journal: Stem Cells Int.

## 3. Conclusions

In summary, there has been an exponential growth in knowledge related to the inherent regenerative potential of teeth and the biological processes that govern stem cell recruitment, proliferation, and differentiation in the context of pulp injury and repair. Although most regenerative procedures have demonstrated to produce reparative tissues, there is strong evidence that, in these cases, the major components of the pulp-dentin complex are present, such as mineralizing cells, blood vessels, immune cells, innervation, an organized extracellular matrix, and lymphatic vessels [80]. However, there is still the need to have better spatial and temporal control of the tissues formed in a predictable way. More importantly, the clinical outcome of continued root development is not always achieved in correctly applied regenerative therapies. It is expected that the drive to develop methods to best control tissue formation serves as a catalyst for the translation of these methods to the clinical practice that would result in increased predictability for the desired clinical outcomes with the overarching goal of prolonging the longevity of the permanent dentition. As discussed above, there have been clinical trials that utilized cell-based therapies or tissue transplants from donor teeth to promote the functional regeneration of permanent teeth. However, the evidence that these cell-based procedures promote the regeneration of the pulp-dentin complex to its natural histological architecture is extremely limited and only shown in one sample in a recent clinical trial [55]. Nonetheless, this approach allows for better control of the triad of tissue engineering since purified cells or even partially differentiated cells could be used in a specific scaffold with or without the addition of growth factors. Lastly, as the field of regenerative endodontics evolves, the challenges of a biocompatible disinfection, removal of residual toxins, and the control of the hypoxic gradient within a root canal that is initially devoid of vascularity need to be addressed. This review discussed how the microbial challenge of an immature infected tooth and how disinfection strategies can regulate stem cell fate. Also, it is well-established that residual bacterial antigens such as liposaccharide (LPS) persist within the root canals following disinfection and have a robust effect on the differentiation of MSCs. Similarly, cells applied in hypoxic environment have altered differentiation potentials. Therefore, future regenerative therapies must include strategies to best disinfect, detoxify, and regulate hypoxia in order have optimal control of stem cell, proliferation, differentiation, and integration with the microenvironment to fully recapitulate the native pulp-dentin complex in architecture and function and the goal of restoring the permanent dentition.

The article "The Four Pillars for Successful Regenerative Therapy in Endodontics: Stem Cells, Biomaterials, Growth Factors, and Their Synergistic Interactions" was published in 2022. Journal: Stem Cells Int.

Finally, this review specifies that both basic knowledge and practical information are required to warrant the proper translational applications of the emerging technologies in biomaterials and signaling molecules and recent advances in stem cell therapy, in regenerative endodontics. We also provide useful and timely clinical evidence offering dental specialists the tools and knowledge they need for the preservation or reestablishment of tooth vitality and functionality.

## Figures and Tables

**Figure 1:** The four pillars of REPs: 1 Stem cells, CF-RET: exogenous stem cells and CB-RET: exogenous stem cells. 2 Biomaterials: Biological PRP: platelet-rich plasma or PRF: platelet-rich. 3 Growth factors (GF): From dentin walls and blood clot or GF-impregnated scaffold. 4 Synergistic interactions between.

**Table 1:** Comparison between cell-free regenerative endodontic therapy (CF-RET) and cell-based regenerative endodontic therapy (CB-RET).

	CF-RET	CB-RET
Cells	Autologous (endogenous source) Nature unknown Amount unknown	Autologous or allogenic (exogenous source)^∗^ Nature known Amount known
Scaffold	Biological	Biological or synthetic
Growth Factors	Dentin walls or blood clot	Dentin walls or added to the scaffold

^∗^Cells taken out from the host or other donors and cultured in vitro before delivering back to the host.

**Table 2:** *In vivo* and *in vitro* studies reported.

Authors and number of cite	Year	Study design	Stem cells	Scaffold	Bioactive molecules	Most relevant findings
Dissanayaka et al.	2014	In vivo in immunodeficient mice	Dental pulp stem cells (DPSCs) prevascularized by human umbilical vein endothelial cells (HUVECs)	No	No	(i) After four-week implantation, tooth-root slices containing microtissue spheroids resulted in well-vascularized and cellular pulp-like tissues. (ii) Immunohistochemical staining indicated that the tissue found in the tooth-root slices was of human origin. (iii) Vascular structures formed by HUVECs *in vitro* were successfully anastomosed with the host vasculature upon transplantation *in vivo.*

Dissanayaka et al.	2015	In vitro	Dental pulp stem cells (DPSCs) prevascularized by human umbilical vein endothelial cells (HUVECs)	Agarose micromolds	No	(i) DPC microtissue microenvironment supported HUVEC survival and capillary network formation in the absence of a scaffolding material and external angiogenic stimulation. (ii) Immunohistochemical staining for CD31 showed the capillary network formed by HUVECs did sustain, for a prolonged period. (iii) Induced, prevascularized macrotissues showed enhanced differentiation capacity compared with DPC alone macrotissues, as shown by higher osteo-/odontogenic gene expression levels and mineralization.

Dissanayaka et al.	2015	In vivo in severe combined immunodeficient (SCID) mice	Human umbilical vein endothelial cells (HUVECs) and/or dental pulp stem cells (DPSCs)	Peptide hydrogel PuraMatrix^TM^	No	(i) DPSCs increased early vascular network formation by facilitating the migration of HUVECs and by increasing vascular endothelial growth factor (VEGF) expression. (ii) Both the DPSC monoculture and coculture groups exhibited vascularized pulp-like tissue with patches of osteodentin after transplantation in mice. (iii) The cocultured groups exhibited more extracellular matrix, vascularization, and mineralization than the DPSC monocultures in vivo. (iv) The DPSCs play a critical role in initial angiogenesis, whereas coordinated efforts by the HUVECs and DPSCs are required to achieve a balance between extracellular matrix deposition and mineralization.

Li et al.	2016	In vivo with 12 immunocompromised nude mice	Dental pulp stem cells (DPSCs)	Growth factor-loaded nanofibrous microsphere scaffolding system with a nanofibrous poly(l-lactic acid) (PLLA) microsphere	Vascular endothelial growth factor (VEGF)	(i) This hierarchical microsphere system not only protects the VEGF from denaturation and degradation but also provides excellent control of its sustained release. (ii) Nanofibrous PLLA microsphere integrates the extracellular matrix-mimicking architecture with a highly porous injectable form, efficiently accommodating dental pulp stem cells (DPSCs) and supporting their proliferation and pulp tissue formation. (iii) Successful regeneration of pulp-like tissues fulfilled the entire apical and middle thirds and reached the coronal third of the full-length root canal. (iv) A large number of blood vessels were regenerated throughout the canal.

Rufas et al.	2016	In vitro	Dental pulp stem cells (DPSCs)	Minimal essential medium	C3a	(i) Addition of recombinant C3a induced a significant proliferation of fibroblasts and DPSCs. (ii) When subjected to a C3a gradient, DPSCs were mobilized but not specifically recruited, whereas pulp fibroblasts were specifically recruited following a C3a gradient. (iii) C3a is involved in increasing DPSCs and fibroblast proliferation, in mobilizing DPSCs, and in specifically guiding fibroblast recruitment.

Wang et al.	2016	In vitro	Human dental pulp cells (hDPCs)	Polycaprolactone/submicron bioactive glass hybrid composites	Cells were cultured in sterile regular medium, supplemented with 10% fetal bovine serum,100 U/mL penicillin, and 100 mg/mL streptomycin	(i) Crystalline apatite was not precipitated on pure PCL and did not exhibit precipitation. (ii) Surface deposition on PCL/smBG hybrids was thicker than on pure bioactive glass scaffolds at a later stage. (iii) Human dental pulp cells had a significantly higher proliferation rate on the PCL/smBG hybrid than on the bioactive glass and PCL scaffolds. (iv) The integration of smBG into the hybrid scaffold significantly promoted the expression of markers for odontogenic differentiation. (v) More mineralized nodules were generated in the PCL/smBG group than in the other 2 groups.

Yadlapati et al.	2017	In vitro and in vivo with 5 female C57BL/6 mice	Human stem cells from apical papilla (SCAP) and NIH-3T3 mouse fibroblasts	A biodegradable drug-loaded fiber realized by a polydioxanone fiber 50 *μ*m in diameter	Vascular endothelial growth factor (VEGF)	(i) Enzyme-linked immunosorbent assay verified detectable concentrations of released VEGF in solution for 25 days. (ii) No cytotoxicity was observed on stem cells of the apical papilla (SCAP) and mouse fibroblasts treated with VEGF. (iii) VEGF treatment also induced the expression of additional growth factors with roles in tissue and blood vessel formation and neuroprotective function. (iv) Implantation of VF and root fragments filled with VF showed biocompatibility in vivo, promoting new blood vessels and connective tissue formation into the root canal space with negligible inflammation.

Chrepa et al.	2017	In vitro	Stem cells of the apical papilla (SCAP)	Commercially available hyaluronic acid hydrogel (Restylane)	Alpha-minimum essential medium (a-MEM) (supplemented with 10% fetal bovine serum)	(i) Cell encapsulation in either Restylane or Matrigel demonstrated reduced cell viability compared with control. (iii) Cell viability significantly increased in the Restylane group in the course of 3 days, whereas it decreased significantly in the Matrigel group. (iii) Restylane promoted significantly greater alkaline phosphatase activity and upregulation of dentin sialo phosphoprotein, dentin matrix acidic phosphoprotein-1, and matrix extracellular phosphoglycoprotein, compared with control.

Soares et al.	2018	In vitro and in vivo	DPCs	Highly porous NF-PLLA	Simvastatin and nanofibrous poly(l-lactic acid) scaffolds to promote the odontogenic potential of dental pulp cells in an inflammatory environment	(i) Adding simvastatin significantly represses the expression of proinflammatory mediators and also reverted the negative effects of LPS on expression of odontoblastic markers in vitro and in vivo. (ii) DPC/NF-PLLA constructs treated with LPS/simvastatin also led to an increase in vessel-like structures, correlated with increased VEGF expression in both DPSCs and endothelial cells. (iii) Combination of low dosage simvastatin and NF-PLLA minimizes the inflammatory reaction and increases the regenerative potential of resident stem cells.

Itoh et al.	2018	In vitro and in vivo	3D DPSC constructs	No	No external growth factors	(i) Pulp-like tissues with rich blood vessels were formed within the human root canal 6 weeks after implantation. (ii) Histologic analyses revealed that transplanted DPSCs differentiated into odontoblast-like mineralizing cells at sites in contact with dentin. (iii) Human CD31–positive endothelial cells were found at the center of regenerated tissue. (iv) Self-organizing ability of 3D DPSC constructs was active within the pulpless root canal in vivo. (v) Blood vessel–rich pulp-like tissues can be formed with DPSCs without requiring scaffolds or growth factors.

Alqahtani et al.	2018	In vitro and in vivo	Human dental pulp stem cells (HDPSC)	Dental pulp extracellular matrix (DP-ECM)	No external growth factors	(i) Decellularized ECM supports cellular infiltration together with the expression of pulp-dentin and vascular markers (DSP and CD31).

The article "The Four Pillars for Successful Regenerative Therapy in Endodontics: Stem Cells, Biomaterials, Growth Factors, and Their Synergistic Interactions" was published in 2022. Journal: Stem Cells Int.

**Table 3:** Published randomized clinical trials.

Authors and number of cite	Study title	Institution	Sample size (teeth	Age	Etiology/type tooth	Intracanal irrigation	Intracanal medication	Groups	Follow-up time	Radiographic evaluation	Success/survival	Main findings	Vitality test
Brizuela et al.	“Cell-Based Regenerative Endodontics for Treatment of Periapical Lesions: A Randomized, Controlled Phase I/II Clinical Trial”	Centro “Activa Biosilicate Technology™” de Investigación en Biología y Regeneración Oral (CIBRO), Faculty of Dentistry, Universidad de los Andes, Santiago, Chile	36p (36 Mt)	16-58 y	Trauma 96.7% (A) Dens evaginatus 3.3% (A)	25% NaOCl 17% EDTA	Calcium hydroxide	Exp (13p/13t): REP/BC-UC-MSCs in PPP-biodentine Control (13p/13t): RC/GP	6-12 m	2D x-ray and 3D-CBCT	6 m: 94.4% (100%) 12 m: 100% (100%)	No difference between groups except for the anterior posterior healing improved for the exp. group. Increase positives vitality responses for exp group	Cold 56%, hot test 28%, EPT 50% at 12 m
ElSheshtawy et al.	“The Effect of Platelet-Rich Plasma as a Scaffold in Regeneration/Revitalization Endodontics of Immature Permanent Teeth Assessed Using 2-Dimensional”	Department of Endodontics, Faculty of Dentistry, Cairo University, Cairo, Egypt	26p (31 It)	8.3-12.1 y	Trauma 96.7% (A) Dens evaginatus 3.3% (A)	5.25% NaOCl 2.5% NaOCl 17% EDTA	TAP 1:1:1	Exp (13p/13t): PRP/MTA Control (13p/13t): BC/MTA	3-6-9-12 m	2D x-ray and 3D-CBCT	87% (100%)	No difference between groups except for the influence of the diameter of the periapical lesion	100% negative response
Xuan et al.	“Deciduous Autologous Tooth Stem Cells Regenerate Dental Pulp after Implantation into Injured Teeth”	Department of Endodontics, Faculty of Dentistry, Health Sciences University, İstanbul, Turkey MS-State Key Laboratory, School of Stomatology, Fourth Military Medical University, Xi'an, China	36p (36 It)	18-30 y	Trauma 100% (A)	3% NaOCl 5% EDTA	Calcium hydroxide/iodoform	Exp (26t): RET/hDPSC/MTA Control (10t): Apx/Ca(OH)	1-2-3-6-9-12-24 m	2D x-ray and 3D-CBCT	100% (100%)	Significant difference in root length	Negative EPT test at 6 and 12 m but increase blood vessels formation
Ulusoy et al.	“Evaluation of Blood Clot, Platelet-Rich Plasma, Platelet-Rich Fibrin, and Platelet Pellet as Scaffolds in Regenerative Endodontic Treatment: A Prospective Randomized Trial”	Department of Pediatric Dentistry, Hacettepe University, Ankara Hacettepe University, Istanbul Okan University, Turkey Louisiana State University Health Sciences Center, New Orleans, Louisiana	88p (88t)	8-11 y	Trauma 100% (A)	5.25% NaOCl 2.5% NaOCl 17% EDTA	TAP 1:1:1	Exp1 (18t): PRP scaffold Exp2 (17t): PRF scaffold Exp3 (17t): PP scaffold Control (21t): BC scaffold	1-3-6-9-12-15-18 m	2D x-ray	95.6%/100%	There was no statistically significant difference in periapical healing, apical closure, but dentinal wall thickening and root length were significant for the BC group	86% positive response to EPT in all groups
Lin et al.	“Regenerative Endodontics Versus Apexification in Immature Permanent Teeth with Apical Periodontitis: A Prospective Randomized Controlled Study”	Dentistry, Operative Dentistry and Endodontics, Department of Radiology, Department of Medical Statistics and Epidemiology, Sun Yat-sen University, Guangzhou, Guangdong, China Guanghua School of Stomatology, Sun Yat-sen University, Guangzhou	103	6-16 y	Dens evaginatus 67% (P) Trauma 33% (A)	1.5% NaOCl 0.9% saline 17% EDTA	∗TAP 0.1 mg/ml with clindamycin	Exp: 67t REP (21t T-A, 48t DE-P) Control: 34t apex MTA (13t T-A, 21t DE-P)	3-6-9-12 m	2D x-ray and 3D-CBCT	RET 89.8% (100%) Apex MTA 97% (100%)	There was statistically significant difference in success rate for the RET group between the DE and trauma cases. The etiology is considered an important factor for success	N/A
Jiang et al.	“Clinical and Radiographic Assessment of the Efficacy of a Collagen Membrane in Regenerative Endodontics: A Randomized, Controlled Clinical Trial”	Department of Pediatric Dentistry, Peking University School and Hospital of Stomatology, Beijing, China	40p (43t)	8.3-12.1y	Trauma 24% (A) Dens evaginatus 76% (P)	1.5% NaOCl 17% EDTA	Calcium hydroxide	Exp (20p/22t): Bio-Gide collagen membrane at mid root/MTA Control (20p/21t): no membrane/MTA	6 months	2D x-ray	100%	No difference between groups except for the increase in the mid third wall thickness on experimental group	Experiment group 33% (+ EPT) Control group 18% (+ EPT)
Bezgin et al.	“Efficacy of Platelet-Rich Plasma as a Scaffold in Regenerative Endodontic Treatment”	Department of Pedodontics, Faculty of Dentistry, Ankara University, Ankara, Turkey	20p (22t)	7-13 y	Trauma 70% (A) Caries 30% (P)	2.5% NaOCl 0.12% CHX 5% EDTA Sterile saline	∗TAP 1:1:1 with cefaclor	Exp (11t): PRP scaffold Control (11t): BC scaffold	1-3-6-9-12-15-18 m	2D x-ray	95.6%/100%	There was no statistically significant difference in periapical healing, apical closure, but dentinal wall thickening between groups	Experiment group 50% (+ EPT and + cold) Control group 20% (+ EPT and cold test)
Nagata et al.	“Traumatized Immature Teeth Treated with 2 Protocols of Pulp Revascularization”	Department of Restorative Dentistry, Endodontics Area, State University of Campinas-UNICAMP, Piracicaba, São Paulo, Brazil	23p (23t)	7-17 y	Trauma 100% (A)	6% NaOCl 5% sodium thiosulfate 2% chlorhexidine 17% EDTA 5% Tween 80 0.07% soy lecithin	CHP 2% or TAP 1:1:1	Exp (11p/11t): CHP calcium hydroxide and 2% chlorhexidine Control (12p/12t): TAP	1-3-6-9-12-15-19 m	2D x-ray	95.6%/100%	There was no statistically significant difference in periapical healing, apical closure, and dentinal wall thickening between groups but CHP show less discoloration	In both groups no recovery of sensitivity
Nagy et al.	“Regenerative Potential of Immature Permanent Teeth with Necrotic Pulps after Different Regenerative Protocols”	Department of Endodontics, Faculty of Dentistry, Ain Shams University, Cairo, Egypt	36p (36t)	9-13 y	N/A, 100% (A)	2.6% NaOCl	TAP 1:1:1	Exp (12p/12t): hydrogel bFGF Control (12p/12t): blood clot Control (12p/12t): MTA apical plug	3-6-12-18 m	2D x-ray	80%/100%	There was no statistically significant difference in periapical healing, apical closure, and dentinal wall thickening	N/A
Jadhav et al.	“Revascularization with and without Platelet-Rich Plasma in Nonvital, Immature, Anterior Teeth: A Pilot Clinical Study”	Department of Conservative Dentistry and Endodontics, Institute of Medical Sciences, New Delhi, India	20p (20t)	15-28 y	N/A	2.5% NaOCl	TAP 1:1:1	Exp (10p/10t): PRP and metronidazole collagen (Metrogene) Control (10p/10t): blood clot	6-12 m	2D x-ray	100%/80%	There was a statistically significant difference in periapical healing, apical closure, and dentinal wall thickening	N/A
